RETRACTED

# Use of Post-Mortem Computed Tomography During the COVID-19 Pandemic: The Malaysian Experience

**DOI:** 10.21315/mjms2022.29.5.9

**Published:** 2022-10-28

**Authors:** Mansharan Kaur Chainchel Singh, Mohamad Helmee Mohd Noor, Mohamad Azaini Ibrahim, Sheue Feng Siew, Poh Soon Lai

**Affiliations:** 1 Institute of Pathology, Laboratory and Forensic Medicine (I-PPerForM), Universiti Teknologi MARA (UiTM), Selangor, Malaysia; 2 Faculty of Medicine, Universiti Teknologi MARA (UiTM), Selangor, Malaysia; 3 National Institute of Forensic Medicine, Hospital Kuala Lumpur, Kuala Lumpur, Malaysia; 4 Radiology Department, Hospital Kuala Lumpur, Kuala Lumpur, Malaysia

**Keywords:** post-mortem computed tomography, COVID-19, autopsy, complement, pandemic

## Abstract

**Background:**

COVID-19 was declared a pandemic by the World Health Organization (WHO). COVID-19 is highly contagious, making it a threat to healthcare workers, including those working in mortuaries. Therefore, it is important to determine if the cause of death (COD) could be identified using limited autopsy, diagnostic tests and post-mortem imaging modalities instead of full autopsy. This study aims to examine the effectiveness of post-mortem imaging, specifically post-mortem computed tomography (PMCT) at determining the COD during a pandemic.

**Methods:**

This cross-sectional study included 172 subjects with suspected or unknown COVID-19 status brought in dead to the institute’s mortuary during the pandemic in Malaysia. PMCT images reported by forensic radiologists and their agreement with conventional autopsy findings by forensic pathologists regarding COD were analysed to look at the effectiveness of PMCT in determining COD during a pandemic.

**Results:**

Analysis showed that 78.7% (133) of cases reported by forensic radiologists concurred with the COD certified by forensic pathologists. Of these cases, 85 (63.9%) had undergone only external examination and real-time reverse transcriptase polymerase chain reaction (rRT-PCR) COVID-19 testing, meaning that imaging was the sole method used to determine the COD besides history from available medical records and the investigating police officer.

**Conclusion:**

PMCT can be used as a complement to medicolegal autopsies in pandemic contexts, as it provides significant information on the possible COD without jeopardising the safety of mortuary health care workers.

## Introduction

In December 2019, cases of pneumonia of unknown cause emerged in Wuhan, Hubei, China, linked to a local seafood wholesale market where poultry, snakes, bats and other live animals were sold illegally. The cause of these pneumonia cases was ultimately found to be a new severe acute respiratory syndrome coronavirus 2 (SARS-CoV-2). In February 2020, the disease caused by this virus was named coronavirus disease 2019 (COVID-19) by the World Health Organization (WHO) and declared a global public health emergency (1–3). This disease had spread to a total of 213 countries across the world, with WHO declaring it a pandemic in March 2020.

RETRACTED

The coronavirus family comprises several zoonotic, enveloped, non-segmented, positive-sense single-stranded RNA viruses that cause serious diseases in humans, including Middle East respiratory syndrome (MERS) and severe acute respiratory syndrome (SARS) (4, 5). Transmission of COVID-19 occurs through droplets produced when speaking, coughing or sneezing and patients present with symptoms of fever, cough and difficulty in breathing, though some may be asymptomatic (1, 2, 6–8).

As a result of the high mortality rate associated with this disease, the Royal College of Pathologists (RCPath) has released guidelines on autopsy for mortuary workers in suspected COVID-19 cases, as have many countries. Malaysia has its own guidelines for handling dead bodies of suspected, probable and confirmed COVID-19 cases (Interim Guidelines Annex 20). These guidelines are important, as the virus causing this disease had been categorised as a hazard group 3 (HG3) organism. The Health and Safety Executive’s (HSE) Advisory Committee on Dangerous Pathogens (ACDP) has categorised pathogens according to four hazard groups (groups 1–4) on the basis of pathogenicity to humans, risk to laboratory workers, transmissibility to the community and whether effective prophylaxis is available. HG3 organisms are defined as those that cause serious disease in humans, constituting a risk to health professionals as they spread in the community; however, effective prophylactic measures against them are available (4, 6, 7).

Infections pose a constant threat to forensic experts working on the deceased and this infection is no exception. Therefore, it is of the utmost importance during this pandemic to determine whether the COD can be identified using external examination, limited autopsy and diagnostic tests with the help of post-mortem imaging modalities instead of through a full conventional autopsy to reduce the mortuary health care workers’ risk of COVID-19 (4, 7).

Forensic imaging, methods of which include post-mortem computed tomography (PMCT), magnetic resonance imaging (MRI) and ultrasound, allows for the non-invasive or minimally invasive detection of findings that may or may not be visible during classical autopsy (9–11). It has been used for more than a century as a complement to medicolegal autopsies and has become an integrated procedure for autopsy investigations in many forensic centres around the world because of its rapid, non-invasive ability to provide permanent documentation of the exact in situ state of body organs (9, 12–14). Prior to the COVID-19 pandemic, death certification at the National Institute of Forensic Medicine was confirmed based on the gold standard of gross examination during autopsy, as well as complementary laboratory investigations and PMCT findings.

RETRACTED

This manuscript aims to highlight how the institute’s protocol was adapted during the pandemic, as autopsies were no longer routinely being performed, as well as the effectiveness of PMCT as an adjunct to conventional autopsy in determining the cause of death (COD) which would reduce healthcare workers’ risk of COVID-19 infection.

## Methods

Malaysia imposed a strict lockdown starting 18 March 2020 when the daily number of cases rose above 100 and the number of deaths was increasing. Because the virus causing this disease had been categorised as a HG3 organism, conventional autopsy was considered to be high risk and the number of autopsies performed reduced. Furthermore, the vast majority of the deceased brought to the institute did not have typical signs and symptoms of COVID-19, had inadequate or inaccurate records of possible COVID-19 infection and had no swab tests done prior to death, making conventional autopsies even riskier. During the pandemic, the process of death certification at the institute has relied heavily on PMCT, as the performance of full autopsies and detailed histopathological examinations has been limited. This made the use of PMCT extremely helpful in determining the COD.

All brought in dead (BID) cases to the emergency department or to the institute by the police with a request for post-mortem examination between 18 March 2020 and 9 June 2020, during the peak of the second wave of the pandemic, were included in this study based on convenience sampling. However, 22 cases that that did not undergo a PMCT scan were excluded.

### Post-Mortem Chest Computed Tomography Scan Imaging

A new workflow was set up at the institute to handle cases during the pandemic, as shown in Figure 1. PMCT scans were performed only once daily in the morning, unlike previously, when scans were performed within 6 h of the deceased’s arrival to the institute. This was to reduce the time spent donning and doffing appropriate personal protective equipment and clothing (N95 or N100 masks, long-sleeved fluid-repellent disposable gowns and gloves) worn by staff handling the deceased. Each deceased was placed in a two-layer body bag and a native PMCT scan was performed prior to any manipulation of the body using a 64-slice (Toshiba Aquilion 64 TSX-101A, Japan) multi-detector computed tomography (MDCT) scanner, a machine wholly dedicated to use in autopsies. Examinations were performed in a cranio-caudal direction from head to toe using 1 mm slice thickness for the head region and 2 mm slice thickness for the thorax, abdomen, pelvis and down to the toes. The following pre-defined scanning protocols were used: 120 kVp, auto set mAs (Caredose), FOV 500 (LL), 1.0 × 32 raw detector collimation and 0.844/standard pitch.

RETRACTED

PMCT reporting was completed following predefined protocols implemented at the institute by two qualified forensic radiologists with more than 5 years’ experience each. Reporting was conducted by examining the whole body with particular attention to the respiratory system, especially for cases who died naturally, to help forensic pathologists determine the COD and, if possible, diagnose COVID-19 infection. Living patients diagnosed with COVID-19 infection were previously found to have typical chest computed tomography (CT) findings, such as ground glass opacities (GGO), consolidation and traction bronchiectasis (1, 2, 15, 16). Thus, similar chest findings were used to identify this infection via PMCT at our institute, as described by the University of New Mexico (17) (Figures 2a and 2b).

### Autopsy

Autopsy, a post-mortem examination to determine the COD, comprises external and internal examinations, including medicolegal specimen sampling. A full autopsy includes a detailed external examination of the entire body and an internal examination, which involves the removal and dissection of the brain, neck and all thoraco-abdominal organs. A limited autopsy comprises only an internal examination, with medicolegal specimen sampling limited to certain areas of the body.

Autopsies were performed on the cases included in the present study by forensic pathologists with the assistance of medical officers and trained forensic pathology technicians. The autopsies were performed in a negative-pressure autopsy suite of biosafety level 3 in accordance with the interim guidelines of the institute, similar to those followed in other institutions (18–20). Nasopharyngeal swabs were also taken, placed in transport media and sent to the hospital laboratory, where real-time reverse transcriptase polymerase chain reaction (rRT-PCR) testing was performed in cases with suspected COVID-19 infection.

### Statistical Analysis

Demographic data were collected for all autopsy cases received at the institute during the study period. Descriptive statistics based on gender, age and ethnicity or nationality were captured during the study period for all cases that underwent autopsy, whether limited or full, and/or sample-taking with concurrent PMCT imaging. The percentage of cases for which limited autopsy, full autopsy and sample–taking for diagnostic tests were interpreted in this study, as was the percentage of agreement between radiology reports and certified COD.

RETRACTED

## Results

A total of 194 cases were brought to the institute during the period between the Movement Control Order (MCO) and Conditional Movement Control Order (CMCO). However, 22 cases did not undergo CT scanning because the CT scanner was not functioning, resulting in a total of 172 cases. Of the 172 cases scanned, 137 (79.7%) were males and the remaining 35 (20.3%) were females (Table 1). This ratio was consistent with the annual gender ratio of 4:1 (male:female) of autopsy cases. The majority of cases in this study were within the age range of 30 years old– 59 years old (59.9%, 103/172) with an average age of 45.6 ± 19.6 years old. A total of 106 (61.63%) cases were Malaysian, with the majority being of Malay descent (52.8%), followed by Chinese (34.0%) and Indian (11.3%) descent. This ethnic distribution correlates with that of the general Malaysian population. Other nationalities (61 cases) included Southeast Asians (42.4%) and other Asian groups (42.4%).

Out of the 172 autopsy cases that underwent PMCT scans, external examination was performed in 77 cases (44.8%), with blood and urine samples taken for further investigation, without a full autopsy examination (Table 2). Thus, these cases relied heavily on post-mortem CT findings reported by forensic radiologists to determine COD. Full or limited autopsy was performed in 73 PMCT-scanned cases (42.4%), with tissue taken for histopathology examination and, in some decomposed cases, toxicology analysis. In another 21 PMCT-scanned cases (12.2%), only external examination was conducted and respiratory swabs for rRT-PCR COVID-19 testing taken, with neither dissection nor sample-taking. All these cases were reviewed by certified forensic radiologists, who then determined the COD which was certified by the forensic medical officer or forensic medicine specialist after discussion and with reference to the CT scan findings. Only one case (0.6%), a road traffic accident case, was managed solely using PMCT findings, with neither dissection nor sample-taking. The injuries in this case were documented externally and PMCT images were reviewed by a forensic radiologist.

A total of 154 respiratory swabs (90.7%) were taken for rRT-PCR COVID-19, testing as most BID cases were flagged as persons under investigation (PUI) for COVID-19 infection during the study period or had suspicious lung findings on the PMCT scan. However, only one of these cases tested positive for COVID-19. Findings that indicated suspicion for COVID-19 were those with GGO, lung consolidation, crazy paving pattern and traction bronchiectasis. Triage according to this imaging was found to be useful in alerting the forensic pathologist to a possible COVID-19 infection, thereby improving the workflow and safety of those involved. The Spearman’s rank correlation coefficient for pneumonia findings from PMCT reports as compared to rRT-PCR testing was relatively low at *r* = 0.144, *P* > 0.05. This shows that rRT-PCR will remain the gold standard for COVID-19 infection while PMCT should be used only as a screening tool for COVID-19 diagnosis.

RETRACTED

## Discussion

As the number of active positive COVID-19 cases in Malaysia continued to rise, the institute had to prepare for an increase in the number of deaths due to COVID-19, which had the potential to overwhelm the capacity of the forensic service. Thus, the institute improvised procedures and guidelines to manage the dead within existing regulations to achieve a balance between medicolegal requirements and the safety of personnel managing bodies with suspected or confirmed COVID-19 infection (19). These protocols included performing rRT-PCR to confirm COVID-19 infection, as well as the use of imaging (i.e. PMCT) to assist in determining the COD in possible COVID-19 cases, as autopsies were in decline during this pandemic.

At the institute, out of 154 cases with PMCT reports of respiratory findings for which swabs were taken, only 34 cases had pneumonia-related certified CODs, including one positive COVID-19 case. Thus, PMCT over-diagnosed findings of pneumonia, raising the possibility of COVID-19 infection and necessitating swabs to be taken for the gold-standard rRT-PCR test. In other words, PMCT accurately diagnosed COVID-19 in one case but raised suspicion of respiratory cases as a COD in 22.1% of cases, for which the Spearman’s rank correlation coefficient was reported at *r* = 0.590, *P* < 0.001. In the rest (77.3%) of the cases, COD was related to cardiac pathology, head and/or neck injuries and pathology in other organs. The distribution of the various types of COD encountered during this period is illustrated in Table 3.

CT is used extensively in the diagnosis of COVID-19-infected patients as it is easy to perform, provides data rapidly and is relatively sensitive for diagnosis (1, 2, 15, 16). However, as with any diagnostic tool, there is a potential for false negative detection because CT findings can mimic pneumonia. It has been reported that in the early stages of some infections, CT may appear almost normal (17). Furthermore, the characteristic findings of COVID-19 on CT are described as GGO, which may evolve to consolidations. These are commonly seen in dependent parts of the lungs as part of post-mortem changes even before the pandemic, which makes it difficult at times to diagnose COVID-19 infection.

RETRACTED

The correlation between PMCT findings and certified CODs was evaluated by an independent specialist in this study. COD was determined by forensic medical officers and specialists based on history and autopsy, while COD was determined by forensic radiologists based solely on PMCT imaging findings. Among the 172 cases selected in this study, the forensic radiologists reported CODs that concurred with the CODs certified by the forensic medical officers and specialists in 78.7% (133) cases. Of these 133 cases, 85 (63.9%) underwent only external examination and rRT-PCR COVID-19 testing. In such cases, forensic radiology services played an important role in determining COD while reducing the risk of infection to healthcare workers. This is in accordance with previous literature, which has shown that PMCT also provided significant information and showed significant accuracy in terms of death categorisation in reference to the final COD category (21, 22).

The range of agreement between radiology findings reported by the forensic radiologists and COD certified by the forensic medical officers and medicine specialists was 90.0% for undetermined COD and decomposed bodies, 87.9% for respiratory-related deaths, 80.2% for heart- or cardiac-related deaths, 74.1% for brain-related deaths and 37.5% for COD in other organs (Figure 3).

Therefore, with all its limitations, PMCT still proved to be a good diagnostic tool during the pandemic. The benefit of using PMCT was to reduce the risk of contracting life-threatening infectious disease (i.e. COVID-19) while performing conventional autopsy, as it allowed for additional precautions to be taken and appropriate personal protective equipment to be worn by personnel prior to autopsy without the need for a confirmed COVID-19 diagnosis. Comparison was made between PMCT and autopsy results by looking at the identified COD rather than the ability to diagnose COVID-19 (23) because CT findings associated with COVID-19 are known to be non-specific. Thus far, there have been no incidents of COVID-19 infection reported within the forensic fraternity at our institute during this period.

## Conclusion

Although post-mortem CT was not found to be superior to molecular testing at the laboratory for COVID-19 diagnosis, forensic radiologists at the institute modulated their protocol during this pandemic to adapt to the risk of COVID-19 and their reports have been beneficial in assisting the forensic medical officer and specialists in the certification of COD. Virtual autopsy with a standardised triage criterion internationally agreed upon by forensic radiologists will be the way forward in the future, to determine COD especially during pandemics. In summary, forensic radiology has once again proven to be complementary to conventional forensic autopsy and will continue to evolve to remain current with the changing landscape of forensic practice.

RETRACTED

## Figures and Tables

**Figure 1:** Flow chart for PMCT examination of suspected or probable COVID-19 cases brought to IPFN

**Figure 2a:** Axial PMCT scan of the chest showing ground glass opacities (blue arrow) and consolidation (red arrow)

**Figure 2b:** Coronal PMCT scan of the chest showing consolidation (red arrow)

**Figure 3:** Percentage of agreement between radiology report and certified COD

**Table 1:** Distribution of post-mortem cases with a PMCT scan according to gender, age and ethnicity or nationality

	Number of cases (%) (*N* = 172)
Gender	
Male	137 (79.7)
Female	35 (20.3)
Age (years old)	
0–9	10 (5.8)
10–19	1 (0.6)
20–29	17 (9.9)
30–39	29 (16.9)
40–49	43 (25.0)
50–59	30 (17.4)
60–69	21 (12.2)
70–79	12 (7.0)
80–89	3 (1.7)
90–99	2 (1.2)
Unknown	4 (2.3)
Ethnicity/Nationality	
Malay	56 (32.6)
Chinese	36 (20.9)
Indian	12 (7.0)
Other Malaysian	2 (1.2)
Foreigner	61 (35.4)
Unknown	5 (2.9)

**Table 2:** PMCT cases with different autopsy approaches

No.	Description	Number of cases (%)
i.	External examination with blood and/or urine sampling	77 (44.8)
ii.	Full or limited autopsy with histopathological sampling	73 (42.4)
iii.	External examination	21 (12.2)
iv.	Solely on PMCT	1 (0.6)

**Table 3:** Autopsy cases based on COD

Types of cause of death	Number of cases
Cardiac	96
Respiratory	61
Head/Neck/Brain	34
Others	12
Undetermined/Decomposed	11

## References

[1] Zhao W, Zhong Z, Xie X, Yu Q, Liu J (2020). Relation between chest CT findings and clinical conditions of coronavirus disease (COVID-19) pneumonia: a multicenter study. Am J Roentgenol.

[2] Hu L, Wang C (2020). Radiological role in the detection, diagnosis and monitoring for the coronavirus disease 2019 (COVID-19). Eur Rev Med Pharmacol Sci.

[3] Fitzek A, Sperhake J, Edler C, Schröder A, Heinemann A, Heinrich F (2020). Evidence for systematic autopsies in COVID-19 positive deceased: case report of the first German investigated COVID-19 death. Rechtsmedizin (Berl).

[4] Hanley B, Lucas SB, Youd E, Swift B, Osborn M (2020). Autopsy in suspected COVID-19 cases. J Clin Pathol.

[5] Barton LM, Duval EJ, Stroberg E, Ghosh S, Mukhopadhyay S (2020). COVID-19 autopsies, Oklahoma, USA. Am J Clin Pathol.

RETRACTED

[6] Fineschi V, Aprile A, Aquila I, Arcangeli M, Asmundo A, Bacci M (2020). Management of the corpse with suspect, probable or confirmed COVID-19 respiratory infection—Italian interim recommendations for personnel potentially exposed to material from corpses, including body fluids, in morgue structures, during autopsy practice. Pathologica.

[7] Keten D, Okdemir E, Keten A (2020). Precautions in postmortem examinations in COVID-19-related deaths: recommendations from Germany. J Forensic Leg Med.

[8] World Health Organization (WHO) (2020). Infection prevention and control for the safe management of a dead body in the context of COVID-19.

[9] Thali MJ, Jackowski C, Oesterhelweg L, Ross SG, Dirnhofer R (2007). VIRTOPSY–the Swiss virtual autopsy approach. Leg Med.

[10] 1O’Donnell C, Woodford N (2008). Post-mortem radiology—a new sub-speciality?. Clin Radiol.

[11] Leth PM, Thomsen J (2013). Experience with post-mortem computed tomography in Southern Denmark 2006–11. J Forensic Radiol Imaging.

[12] Grabherr S, Baumann P, Minoiu C, Fahrni S, Mangin P (2016). Post-mortem imaging in forensic investigations: current utility, limitations, and ongoing developments. Res Reports Forensic Med Sci.

[13] Eriksson A, Gustafsson T, Höistad M, Hultcrantz M, Jacobson S, Mejare I (2017). Diagnostic accuracy of postmortem imaging vs autopsy—a systematic review. Eur J Radiol.

[14] Beck JJ (2011). What is the future of imaging in forensic practice?. Radiography.

[15] Fang Y, Zhang H, Xie J, Lin M, Ying L, Pang P (2020). Sensitivity of chest CT for COVID-19: comparison to RT-PCR. Radiology.

[16] Schweitzer W, Ruder T, Baumeister R, Bolliger S, Thali M, Meixner E (2020). Implications for forensic death investigations from first Swiss case of non-hospital treatment with COVID-19. Forensic Imaging.

[17] Helmrich E, Decker L, Adolphi N, Makino Y (2020). Post-mortem CT lung findings in decedents with COVID-19: a review of 14 decedents and potential triage implications. Forensic Imaging.

[18] Lacy JM, Brooks EG, Akers J, Armstrong D, Decker L, Gonzalez A (2020). COVID-19: post-mortem diagnostic and biosafety considerations. Am J Forensic Med Pathol.

[19] Khoo LS, Hasmi AH, Ibrahim MA, Mahmood MS (2020). Management of the dead during COVID-19 outbreak in Malaysia. Forensic Sci Med Pathol.

[20] Hasmi AH, Khoo LS, Koo ZP, Suriani MUA, Hamdan AN, Yaro SWM (2020). The craniotomy box: an innovative method of containing hazardous aerosols generated during skull saw use in autopsy on a COVID-19 body. Forensic Sci Med Pathol.

[21] Ampanozi G, Thali YA, Schweitzer W, Hatch GM, Ebert LC, Thali MJ (2017). Accuracy of non-contrast PMCT for determining COD. Forensic Sci Med Pathol.

RETRACTED

[22] Roberts IS, Benamore RE, Benbow EW, Lee SH, Harris JN, Jackson A (2012). Post-mortem imaging as an alternative to autopsy in the diagnosis of adult deaths: a validation study. Lancet.

[23] Malizia A, Filograna L, Ryan C, Manenti G (2020). Post-mortem investigation through virtual autopsy techniques: proposal of a new diagnostic approach to reduce the risks of operators during emergencies. Int J Safety Security Engineer.

